The article "Xiaotan Sanjie Decoction Inhibits Gastric Cancer Cell Proliferation, Migration, and Invasion through lncRNA-ATB and miR-200A" was published in 2022. Journal: Biomed Res Int.

# Xiaotan Sanjie Decoction Inhibits Gastric Cancer Cell Proliferation, Migration, and Invasion through lncRNA-ATB and miR-200A

**DOI:** 10.1155/2022/7029182

**Published:** 2022-08-25

**Authors:** Zhe Zhou, Jiabin Chen, Mingqian Li, Liping Cao, Miao Chen, Qingqian Zhang, Zhihong Yu, Kequn Chai

**Affiliations:** ^1^The Second Clinical Medical College, Zhejiang Chinese Medicine University, Hangzhou 310053, Zhejiang Province, China; ^2^Cancer Institute of Integrated Tradition Chinese and Western Medicine, Zhejiang Academy of Traditional Chinese Medicine, Tongde Hospital of Zhejiang Province, Hangzhou 310012, Zhejiang Province, China; ^3^Zhejiang Provincial Key Laboratory of Cancer Prevention and Treatment Technology of Integrated Traditional Chinese and Western Medicine, Hangzhou 310012, Zhejiang Province, China

## Abstract

This study is aimed at exploring whether Xiaotan Sanjie decoction (XTSJ) inhibits gastric cancer (GC) proliferation and metastasis by regulating lncRNA-ATB expression. qRT-PCR and Western blot were used to analyze lncRNA-ATB and downstream-regulated genes/proteins in human GC cells. CCK8, Edu, and flow cytometry assays were used to detect the inhibitory effect of XTSJ on cell proliferation and apoptosis. Moreover, transwell and wound healing assays were used to detect the inhibitory effect of XTSJ on migration and invasion. qRT-PCR and Western blot were used to detect regulated genes and proteins levels. The HGC-27 cell line was used for follow-up analysis due to the high level of lncRNA-ATB and cell characteristics. XTSJ inhibited the proliferation and metastasis of HGC-27 in a dose-dependent manner. Further research found that XTSJ downregulated lncRNA-ATB, Vimentin, and N-cadherin, while it upregulated miR-200a and E-cadherin in a dose-dependent manner. XTSJ also upregulated Caspase 3, Caspase 9, Bax, and downregulated Bcl-2. Furthermore, XTSJ inhibited tumor growth *in vivo* and downregulated EMT signaling pathways. These results indicate that XTSJ may affect EMT and Bcl-2 signaling pathways by regulating lncRNA-ATB and miR-200a, thus inhibiting proliferation, migration, and invasion of HGC-27 cells. Therefore, XTSJ may be an effective treatment for the high levels of lncRNA-ATB in GC.

## 1. Introduction

Gastric cancer (GC) has a poor prognosis and is the leading cause of cancer-related deaths [1]. Research has shown that traditional Chinese medicine can treat cancer [2, 3]. Therefore, studying the molecular pathways of traditional Chinese medicine can effectively enhance GC treatment.

lncRNAs are long-chain noncoding RNAs regulating gene transcription and downstream biological signals in tumors [4, 5]. Preliminarily studies have shown that lncRNAs acts as “sponge” to modulate downstream biological signals by competitively binding or chelating microRNAs [6]. TGF-*β*-activated lncRNA-ATB can enhance epithelial-mesenchymal transition(EMT)-related metastasis and proliferation by competitively binding to the miR-200 family in certain malignant tumors [7, 8]. Recent research showed that lncRNA-ATB upregulation in GC enhances vascular infiltration and overall survival while lncRNA-ATB silencing inhibits cell proliferation [9]. Therefore, lncRNA-ATB and miR-200a are potential therapeutic targets for GC treatment.

The article "Xiaotan Sanjie Decoction Inhibits Gastric Cancer Cell Proliferation, Migration, and Invasion through lncRNA-ATB and miR-200A" was published in 2022. Journal: Biomed Res Int.

Xiaotan Sanjie decoction (XTSJ) can effectively prolong the survival of GC patients, decrease TGF-*β* and IL-8 levels, and inhibit the expression of fibroblast activation protein (FAP) [10, 11]. This research aimed to assess whether XTSJ prevents GC proliferation and metastasis by regulating lncRNA-ATB and miR-200a.

## 2. Material and Methods

### 2.1. Cell Culture

MKN-45, SNU-1, HGC-27, AGS, and MGC-803 were obtained from the Institute of Biochemistry and Cell Biology at the Chinese Academy of Sciences. The cells were cultured in RPMI-1640 medium with 10% fetal bovine serum (ExCell bio, Shanghai, China).

### 2.2. Preparation of Drugs

Prof. Wei Pinkang provided the XTSJ. XTSJ components have been described in previous papers. Its active components have been analyzed via HPLC [12]. The 5-fluorouracil (5-Fu) was obtained from Lilly France (Suzhou, China).

### 2.3. CCK-8 Assay

The GC cells (5 × 10^3^ cells/well) were reinoculated and treated with XTSJ for 24, 48, and 72 hours. An appropriate amount of CCK-8 solution was added to the sample, then incubated for 2 hours. A SpectraMax i3 microplate reader (Molecular Devices, CA, USA) was used to measure absorbance.

### 2.4. Ethynyl-2-Deoxyuridine (EdU) Assay

The HGC-27 cells (5 × 10^3^ cells/well) were reinoculated and treated with XTSJ for 24 hours. EdU (100 *μ*L; 50 *μ* m) was then added to the sample then co-cultured for 2 hours. Hoechst3342 (5 *μ*g/ml) was stained at room temperature for 20 minutes. An Olympus TH4-200 fluorescence microscope (Olympus, Tokyo, Japan) was used to obtain images.

### 2.5. Flow Cytometry Assay

The HGC-27 cells (4 × 10^5^ cells/well) were treated with Annexin V-fluorescein isothiocyanate and propidium iodide (Procell, Wuhan, China) for 15 minutes under a shading environment. BD FACSCanto™ II Flow Cytometry System (BD Biosciences, NJ, USA) was used to detect cell apoptosis.

### 2.6. Transwell Migration and Invasion Assays

The HGC-27 cells (4 × 10^4^ cells/well) were reinoculated into the upper chamber coated with Matrigel for invasion assay. For the migration assay, HGC-27 cells (4 × 10^4^ cells/well) were reinoculated into the upper chamber (4 × 10^4^ cells/well) without Matrigel. The upper chamber was filled with serum-free medium, while the lower chamber was filled with medium containing 10% FBS. The transwell chambers were fixed with a 4.0% paraformaldehyde solution for 15 minutes, then stained with a 0.1% crystal violet solution for 10 minutes. A Leica DMi1 inverted microscope (Leica, Wetzlar, Germany) was used to obtain images.

The article "Xiaotan Sanjie Decoction Inhibits Gastric Cancer Cell Proliferation, Migration, and Invasion through lncRNA-ATB and miR-200A" was published in 2022. Journal: Biomed Res Int.

### 2.7. Wound-Healing Assay

The HGC-27 cells (4 × 10^5^ cells/well) were reinoculated until they reached 90% confluence. A 200 *μ*l sterile pipette tip was then used to scratch the center of each well. A Leica DMi1 inverted microscope was then used to assess the wound after 0, 24, and 48 hours.

### 2.8. Western Blot

Total protein was extracted from the HGC-27 cells (3 × 10^6^ cells/well) cells using cell lysate buffer after 24 hours. BCA protein quantitative Kit (Sangon Biotech, Shanghai, China) was used for protein quantitation. Protein concentration was adjusted before protein denaturation. Electrophoresis of the protein sample was conducted on SDS-polyacrylamide gels at 60 V for 3-5 hours. The samples were then transferred onto polyvinylidene difluoride film (Bio-Rad, Hercules, CA, USA) at 300 mA for 90 minutes. The film was blocked with a 5% BSA solution for 90 minutes, then incubated with primary antibodies (E-cadherin (20874-1-AP), Vimentin (60330-1-lg), N-cadherin (22018-1-AP), ZEB-1 (21544-1-AP), Bcl-2 (26593-1-AP), Bax (50599-2-Ig), Caspase 3 (19677-1-AP), Caspase 9 (10380-1-AP), and *β*-actin (66009-1-lg)) at 4°C overnight. The films were then incubated with secondary antibodies (HRP-conjugated Affinipure Goat Anti-mouse IgG (H + L) (SA00001-1) and HRP-conjugated Affinipure Goat Anti-rabbit IgG (H + L) (SA00001-2)) at room temperature for 60 minutes. These antibodies were obtained from Proteintech™ (Wuhan, China). The proteins were visualized using chemiluminescence. Grayscale analysis of Western blot images was conducted using ImageJ.

### 2.9. Real-Time Quantitative Reverse Transcription PCR (qRT-PCR)

Total RNA was obtained from the HGC-27 (3 × 10^6^ cells/well) cells using Trizol reagent after 24 hours. The RNAs were reverse transcribed using the reverse aid first-strand cDNA synthesis Kit (Thermo Fisher Scientific, Ma, USA) to obtain cDNA. A LightCycler® 480 Real-Time PCR System (Roche, Basel, Switzerland) was used for qRT-PCR analysis. Each sample had three replicates. The primer sequences used for amplification are shown in Table 1. Quantitative analysis of each sample was conducted using the 2^-△△Ct^ method.

### 2.10. *In Vivo* Experiment

BALB/c nude mice (6-week-old, female) were reared in a sterile environment. The animal experiment was approved by the Ethics Committee of the Tongde Hospital of Zhejiang Province. The tumor model was established by subcutaneously inoculating the HGC-27 cells (1 × 10^6^ cells/well) into the right side of mouse back. The mice were treated using intragastric of XTSJ (1 g/kg for low-dose and 2 g/kg for high-dose) or intraperitoneal injection of 5-FU (30 mg/kg) every day. The mice were euthanized after seven days. The tumor tissues were dissected and collected. Pathological examination and SABER-FISH were used to assess the expression of EMT related antibodies and the location of lncRNA-ATB in tissues [13, 14].

The article "Xiaotan Sanjie Decoction Inhibits Gastric Cancer Cell Proliferation, Migration, and Invasion through lncRNA-ATB and miR-200A" was published in 2022. Journal: Biomed Res Int.

### 2.11. Statistical Analysis

Quantitative data are expressed as mean ± SD. The normally distributed data were analyzed using students' *t*-test analyzed. Mann–Whitney *U*-test was used to analyze the nonnormally distributed data. Graph-Pad Prism8. 0 software was used for data analysis and drawing charts. *P* < 0.05, *P* < 0.01, and *P* < 0.001 represent significant differences.

## 3. Results

### 3.1. HGC27 Cell Line as a Model for Drug Intervention of lncRNA-ATB *In Vitro*

lncRNA-ATB and EMT signal pathway-related genes and proteins in five GC cells were analyzed to find a suitable cell model for *in vitro* drug intervention of lncRNA-ATB. lncRNA-ATB, Vimentin, and N-cadherin were upregulated in HGC-27 and MKN-45, while miR-200a and E-cadherin were downregulated (Figure 1(a)). Western blot also revealed that ZEB-1, Vimentin, and N-cadherin were upregulated in HGC-27 while E-cadherin was downregulated (Figure 1(b)). However, ZEB-1, Vimentin, and N-cadherin protein levels were relatively low in MKN-45 (a semisuspended cell), while E-cadherin level was relatively high (Figure 1(b)). Moreover, the viability of cells was detected using CCK8. HGC-27 had the lowest IC50 concentration (0.1354 mg/ml), indicating it was the most sensitive to drugs (Figure 1(c)). As a result, HGC-27 was selected as a model for drug intervention *in vitro*.

### 3.2. XTSJ Inhibits Proliferation and Promotes Apoptosis in HGC-27 Cells

Flow cytometry assays showed that apoptosis increased with increasing drug concentration (0 mg/ml, 30.56%; 0.05 mg/ml, 46.23%; 0.1 mg/ml, 50.23%; 0.15 mg/ml, 67.41%; 0.2 mg/ml, 76.16%; 0.3 mg/ml, 83.83%), especially in early apoptosis (Figures 2(b) and 2(c)). EdU assays indicated that the ratio of EdU/Hoechst33342 decreased with increasing XTSJ concentration (0 mg/ml, 59.60%; 0.05 mg/ml, 50.48%; 0.1 mg/ml, 43.93%; 0.15 mg/ml, 31.89%), thus inhibiting proliferation. CCK8 assay showed that XTSJ had an inhibitory effect in a concentration dependent manner (IC50 = 0.1354 mg/ml) and not time-dependent (Figure 2(a)) (Figures 2(d) and 2(e)). These results suggest that XTSJ can inhibit HGC-27 cell proliferation and promote apoptosis.

The article "Xiaotan Sanjie Decoction Inhibits Gastric Cancer Cell Proliferation, Migration, and Invasion through lncRNA-ATB and miR-200A" was published in 2022. Journal: Biomed Res Int.

### 3.3. XTSJ Inhibits Migration and Invasion in HGC-27 Cells

Transwell assays demonstrated that XTSJ significantly reduced cell number in the migration assays at high concentrations (0.15 mg/ml). XTSJ also significantly reduced cell number in the invasion assays in a dose-dependent effect (Figures 3(a) and 3(b)). Wound healing assays found that XTSJ effectively maintained the wound healing range and inhibited cell invasion (Figures 3(c) and 3(d)). These results suggest that XTSJ can effectively inhibit HGC-27 metastasis.

### 3.4. XTSJ Inhibits the Expression of lncRNA and Related EMT and Bcl-2 Signaling Pathways

lncRNA-ATB and downstream-regulated genes and proteins were analyzed using qRT-PCR and Western blotting to reveal how XTSJ inhibits the proliferation and metastasis of HGC-27. qRT-PCR showed that XTSJ reduced the levels of lncRNA-ATB, Vimentin, and N-cadherin while increasing miR-200a and E-cadherin levels in a dose-dependent effect (Figure 4(a)). Similarly, Western blot assays showed that XTSJ reduced ZEB-1, Vimentin, and N-cadherin levels while increasing E-cadherin levels (Figures 4(b) and 4(c)). Western blot also showed that XTSJ reduced Bcl-2 level while it increased Caspase 3, Caspase 9, and Bax levels (Figures 4(d) and 4(e)). These results suggest that XTSJ affects EMT and Bcl-2 signal pathways by downregulating lncRNA-ATB and upregulating miR-200a.

### 3.5. The Effect of XTSJ on GC *In Vivo*

Pharmacodynamic analysis was conducted using HGC-27 transplanted tumor nude mice model. XTSJ inhibited the transplanted tumors in mice, similar to chemotherapeutic drugs (5-FU) (Figures 5(a) and 5(b)). SABER-FISH results showed that lncRNA-ATB was upregulated in the model group while it was downregulated in XTSJ group (Figure 5(c)). Immunohistochemical (IHC) analysis showed that XTSJ reduced the levels of antibodies, such as Ki67, Vimentin, and N-cadherin, while it increased E-cadherin levels (Figure 5(d)). These results indicate that XTSJ can affect EMT signaling pathway *in vivo* (Figure 6).

## 4. Discussion and Conclusion

Gastric cancer (GC) has a poor prognosis, especially GC cells at low to medium differentiation stages that easily undergo proliferation, migration, invasion, and tumorigenesis [15]. Therefore, studies should assess the biological mechanism of proliferation and metastasis in GC.

lncRNA-ATB (TGF-*β* activated long-chain non-coding RNA) >200 nucleotides is located on chromosome 14, and it is related to the occurrence and progression of tumors [16]. lncRNA-ATB is improperly expressed in several cancers, particularly liver cancer [17], colon cancer [18, 19], pancreatic cancer [20], lung cancer [21, 22], breast cancer [23], and ovarian cancer [24, 25], based on research incorporating clinical correlation. Moreover, lncRNA-ATB is related to the prognosis of malignant tumors, including tumor stage, invasion, and metastasis, which directly or indirectly affect the recurrence and overall survival[26]. lncRNA-ATB is also a promising diagnostic index or an index related to drug resistance in some tumors [26–29].

The article "Xiaotan Sanjie Decoction Inhibits Gastric Cancer Cell Proliferation, Migration, and Invasion through lncRNA-ATB and miR-200A" was published in 2022. Journal: Biomed Res Int.

Similarly, lncRNA-ATB was remarkably expressed in GC cells than in adjacent tissues. Increased lncRNA-ATB increases the infiltration depth, distant metastasis, and late tumor lymph node metastasis, affecting the overall survival of GC patients [30]. lncRNAs may act as sponges by competitively binding to microRNAs (miRNAs), thereby inhibiting the active functions [31]. Moreover, lncRNA-ATB silencing can upregulate miR-200 family and induce apoptosis through Bcl-2/caspase 3 pathway in lung cancer and prostate cancer [7, 21]. lncRNA-ATB can also upregulate ZEB1 and ZEB2 by competitively binding to miR-200 family in various tumors [32, 33], resulting in proliferation, migration, and invasion. However, lncRNA-ATB silencing can significantly inhibit ZEB1 and ZEB2 expression, thus inhibiting cell migration and invasion [17, 34]. These results indicate that lncRNA-ATB can affect EMT by competitively binding with miR-200a, thus promoting tumor metastasis in GC [35, 36]. Type I cadherin (epithelial cadherin and E-cadherin) is transformed into N-cadherin and Vimentin (mainly expressed in mesenchymal cells) during EMT [37]. In this study, HGC-27 was selected for follow-up experiments because it had lower E-cadherin and miR-200a levels and higher lncRNA-ATB, Vimentin, N-cadherin, and ZEB-1 levels. XTSJ has been proven in previous research to suppress proliferation, angiogenesis, invasion, and migration [10, 12, 38, 39]. This might be due to the fact that XTSJ lowers lncRNA-ATB and promotes competitive binding to miR-200a, lowering ZEB-1-mediated EMT and Bcl-2-mediated apoptosis. Reduced levels of Vimentin and N-cadherin associated with a mesenchymal phenotype and increasing levels of E-cadherin associated with an epithelial phenotype defined EMT reversal. However, more research should be conducted to identify the major target and effector chemicals of XTSJ that inhibit lncRNA-ATB expression. Furthermore, no research has demonstrated XTSJ's therapeutic effectiveness or associated biomolecular signals in human GC.

In conclusion, XTSJ may affect EMT and Bcl-2 signaling pathways by regulating lncRNA-ATB and miR-200a, thus inhibiting proliferation, migration, and invasion of HGC-27 cells. Therefore, XTSJ may be an effective treatment for the high level of lncRNA-ATB in GC.

The article "Xiaotan Sanjie Decoction Inhibits Gastric Cancer Cell Proliferation, Migration, and Invasion through lncRNA-ATB and miR-200A" was published in 2022. Journal: Biomed Res Int.

## Figures and Tables

**Figure 1:** |Expression of related genes and protein expression in human gastric cancer cells. (a) qRT-PCR analysis of lncRNA-ATB, Vimentin, E-cadherin, N-cadherin, and miR-200a in 5 gastric cancer cells. (b) Western blotting based detection of ZEB-1, Vimentin, E-cadherin, and N-cadherin in 5 gastric cancer cells. (c) Effect of different concentrations of XTSJ on the cell viability in 5 gastric cancer cell lines. ^∗^*P* < 0.05; ^∗∗^*P* < 0.01; ^∗∗∗^*P* < 0.001.

**Figure 2:** Effects of XTSJ on HGC-27 cells proliferation and apoptosis. (a) Effect of different concentrations of XTSJ in the viability of HGC-27 cells. (b) Effects of XTSJ on cells apoptosis were detected by flow cytometry, and (c) the cell apoptosis rate was quantified. (d) EdU assay was performed to observe cell proliferation intervened by XTSJ; blue-labeled (Hoechst 33324) is the nucleus, green-labeled implies the cells undergoing the proliferation process; and (e) the EdU/Hoechst 33324 ratio was quantified. ^∗^*P* < 0.05; ^∗∗^*P* < 0.01; ^∗∗∗^*P* < 0.001.

**Figure 3:** Effects of XTSJ on HGC-27 cell migration and invasion. (a) Effects of XTSJ on the migration and invasion were detected by Transwell assays, and (b) the Transwell cell number was quantified. (c) Wound healing assays detected effects of different concentrations of XTSJ on the cell migration, and (d) the wound area was quantified. ^∗^*P* < 0.05; ^∗∗^*P* < 0.01; ^∗∗∗^*P* < 0.001.

**Figure 4:** Effects of XTSJ on gastric cancer-related mRNA and protein expression. (a) qRT-PCR analysis of lncRNA-ATB, Vimentin, E-cadherin, N-cadherin, and miR-200a after intervention with XTSJ. (b) Western blotting based on detection of ZEB-1, Vimentin, E-cadherin, and N-cadherin after intervention with XTSJ. (c) The relative protein was carried out with *β*-actin as an internal reference. (d) Western blotting based on detection of Bcl-2, Bax, Caspase 3, and Caspase 9 after intervention with XTSJ. (e) The relative protein was carried out with *β*-actin as an internal reference. ^∗^*P* < 0.05; ^∗∗^*P* < 0.01; ^∗∗∗^*P* < 0.001.

**Figure 5:** Effects of XTSJ on gastric cancer in vivo. (a) The tumor volume sizes after subcutaneous inoculation of HGC-27 cells in each group. (b) Tumors were dissected from each group. (c) The expression of SABER-FISH lncRNA-ATB was detected by SABER-FISH. (d) The expression of Ki67, Vimentin, E-cadherin, and N-cadherin in tumor tissues was analyzed by IHC analysis. ^∗^*P* < 0.05; ^∗∗^*P* < 0.01; ^∗∗∗^*P* < 0.001.

**Figure 6:** Molecular mechanism of XTSJ. The corresponding mechanism may be related to XTSJ reducing LncRNA-ATB and increasing miR-200a competing with it to reduce the expression of downstream ZEB-1 and reverse EMT. The process of reversing EMT showed decreased expression of Vimentin and N-cadherin associated with mesenchymal phenotype and increased E-cadherin expression associated with an epithelial phenotype. In addition, XTSJ could reduce Bcl-2, increase Bax, Caspase 3, and Caspase 9 to induce apoptosis.

The article "Xiaotan Sanjie Decoction Inhibits Gastric Cancer Cell Proliferation, Migration, and Invasion through lncRNA-ATB and miR-200A" was published in 2022. Journal: Biomed Res Int.

**Table 1:** Primer sets used in the real-time PCR and qPCR.

Gene name	Primer
lncRNA-ATB	F: TCTGGCTGAGGCTGGTTGAC
	R: ATCTCTGGGTGCTGGTGAAGG
Vimentin	F: AATCCAAGTTTGCTGACCTCTCTGA
	R: GACTGCACCTGTCTCCGGTACTC
E-cadherin	F: GGGGTCTGTCATGGAAGGTGC
	R: GTAAGCGATGGCGGCATTGTA
N-cadherin	F: CATCATCATCCTGCTTATCCTGT
	R: GCTCTTCTTCTCCTCCACCTTCTT
GAPDH	F: ACACCCACTCCTCCACCTTT
	R: TTACTCCTTGGAGGCCATGT
miR-200a	F: CCTACGCCACAATTAACAAGCC
	R: GCCGTCTAACACTGTCTGGTA
U6	F: CTCGCTTCGGCAGCACA
	R: AACGCTTCACGAATTTGCGT

## Data Availability

The data used to support the findings of this study are included within the article.
